RETRACTED

# Effects of Different Polishing Systems on Surface Roughness and Crystal Structure of Zirconia

**DOI:** 10.1155/2022/5360893

**Published:** 2022-05-09

**Authors:** Cheng Chen, Xiaohua Zeng

**Affiliations:** Department of Stomatology, The First Affiliated Hospital of Xiamen University, Xiamen, China

## Abstract

**Objective:**

Intraoral polishing systems have become an alternative method for reglazing, which is important to prevent or minimize rapid wear of the opposing teeth. To assess the influence of different polishing systems and duration on surface roughness and crystal structure of zirconia was compared, contributing to the preparation and effect improvement of clinical zirconia restorations.

**Methods:**

Forty-eight zirconia specimens with equal size were fabricated by cutting and sintering zirconia discs. Then X-ray diffractometer (XRD) was adopted for examination of the specimens. Six specimens were selected as the grinding-polishing group (GL) after polishing, grinding, and glazing. Then six specimens were randomly selected from the remaining specimens as the grinding-unpolished group (GR) after surface conditioning by dental diamond burs. Subsequently, based on different polishing systems and duration, the rest of specimens were divided into following groups (*n* = 6): Youdent-20s group (Y20), Youdent-40s group (Y40), Youdent-60s group (Y60), Toboom-20s group (T20), Toboom-40s group (T40), and Toboom-60s group (T60). Additionally, a contour graph was applied for assessing the surface roughness of zirconia, scanning electron microscope (SEM) for observing surface topography, and X-ray diffraction analysis (XRD) for determining crystal structure of zirconia.

**Results:**

The GR group had the highest roughness, and the roughness of the specimens polished for 20 s with different polishing systems was significantly higher than those polished for 40 s and 60 s with the same polishing systems. There were no significant difference between the Y20 and T20 groups, while the roughness of the specimens in both Y40 and Y60 groups was significantly higher than that of the T40 and T60 groups. And with the increasing polishing duration, the surface morphology of the specimen was gradually smooth and the morphology was gradually regular. Besides, the surface scratches of the T group were shallower than that of the Y group at the same polishing duration. The peak value of XRD profile of the specimen after grinding and polishing process was consistent with the baseline pattern of that the original specimen.

**Conclusion:**

Glazing can reduce the surface roughness of the specimens. Besides, the polishing effect of Toboom (TOB) system (polishing duration = 60 s) is the best. And different polishing durations of TOB system have no significant effect on the crystal surface structure of the specimen.

RETRACTED

## 1. Introduction

With the advent of digital age chair-side milling and the application of novel fast sintering techniques, the fabrication of dental restorations is more precise and efficient. And the development of long-term, durable, and esthetic dental materials is the main direction of dental restorations for current researches [1]. In recent years, all-ceramic restorations have been widely applied in dentistry due to their excellent esthetic properties, biocompatibility, and wear resistance. Zirconia is a polycrystalline material, which has become the preferred restorations in clinical dentistry because of its good mechanical properties, esthetic properties, and biocompatibility [2–4]. The other polycrystalline materials are glass-based ceramics such as feldspathic ceramics which are used as veneers to cover the metal coping and framework. They are also used in the bilayered, all-ceramic restoration method when the aesthetic is considered a dominant factor. The improved strength of highly filled glass-based ceramics such as leucite- and lithium disilicate-based types is considered for use as inlays and onlays, anterior and posterior crowns, and veneers. In the fabrication of zirconia restorations, although the application of computer-aided design greatly increases the accuracy of restorations, the chairside milling is still required in clinical trials to ensure that the shape and morphology and occlusion of restorations are in line with human requirements.

Due to the high hardness, dental diamond burs are often adopted in clinical practice to adjust and modify the surface of zirconia. However, the application of dental diamond burs causes a significant increase in surface roughness of zirconia [5]. Misaligned sliding and grinding of zirconia disc or dental diamond burs can also bring about changes in crystal structure and the formation of amorphous phase [6]. Increased roughness of restorations can cause mechanical wear, stress concentration, attachment plaque, and so on [7–9]. At present, glazing and polishing are common methods to sooth the surface of restorations after occlusal adjustment. It has also been found that the long-term stability of the enamel layer is poor and may not be maintained for a long time in the functional state [10, 11]. Polishing is the operation commonly applied in clinical practice to smooth the surface of restorations. Specifically, polishing not only removes superfluous material by grinding but also eliminates surface defects caused by grinding. And the abrasive in the polishing materials delivers mechanical energy to the materials, to change the surface roughness [12]. The surface roughness of porcelain restorations is reduced after polishing, which can reduce the wear on the enamel of the jaw [13]. Besides, during the polishing process, the speed, tools, strength, and duration may affect the effect of polishing. In the heat treatment, zirconia is changed from tetragonal phase to monoclinic phase and then to be weaken [14]. However, the effect of polishing treatments with heat produce on zirconia phase transition is currently unknown. In this study, the influence of different polishing systems and duration on surface roughness and crystal structure of zirconia was compared, contributing to the preparation and effect improvement of clinical zirconia restorations.

RETRACTED

## 2. Materials and Methods

### 2.1. Preparation of Specimens

CAD/CAM software (3shape, Denmark) was utilized for the typesetting and design of ST zirconia disc (UPzir Solid Zirconia) (Figure 1(a)). Then, a machine tool (Cradle, China) was adopted for cutting and sintering. Specifically, 48 zirconia specimens with the size of 10 mm × 10 mm × 2 mm was prepared with 7 h sintering at 1500°C in sintering furnace (upfire C1, Upcera, China). After that, one of the zirconia specimens was selected randomly to conduct X-ray diffractometer (XRD) detection. Then, the diffraction pattern was obtained (Figure 1(b)) and acted as the reference image (control).

### 2.2. Treatment of Specimen Surface

The specimens were subjected to surface polishing and glazing operation in the laboratory by the same technician to simulate the surface state of restoration before modification. Then, 6 specimens were selected randomly to be as grinding-polishing group (GL). The remaining specimens were processed using surface grinding using a dental diamond bur for 20 s in a water-cooled state to simulate the clinical occlusal adjustment process, with parallel sample surface as the direction of grinding. After grinding, 6 specimens were selected randomly as the grinding-unpolished group (GR). Subsequently, the rest of the specimens were processed using three-step polishing using Youdent (YOU) and Toboom (TOB) systems (Table 1). Polishing without pressure was applied, and the polishing direction was consistent with the grinding direction. According to different polishing systems and duration, the specimens were divided into following groups (*n* = 6): YOU-20s group (Y20), YOU-40s group (Y40), YOU-60s group (Y60), TOB-20s group (T20), TOB-40s group (T40), and TOB-60s group (T60). Ultrasonic cleaning was performed in distilled water for 30 s. After drying, the specimens were determined.

RETRACTED

### 2.3. Roughness Measurement

A probe surface profilometer (DEKTAK-XT, Bruker, America) was utilized to check surface roughness of specimens, with GB/T1031-2009 as a control [15]. All polished center areas for the specimens were detected, with the grinding direction being perpendicular to the specimens as the detection direction. Three measurements were taken for each specimen. And then, the arithmetic mean value of the 3 measurements was calculated.

### 2.4. SEM Observation

One specimen from each group was randomly selected. After drying, the platinum was sprayed on the surface of the specimens by vacuum coating. Then, a high-resolution field-emission scanning electron microscopy (SEM, SIGMA500, ZEISS, Germany) was utilized to observe surface morphology of the specimens (observation fold: 1000 times).

### 2.5. X-Ray Diffractometer (XRD) Detection

One specimen from each group was randomly selected to detect the surface crystalline structure with XRD (Ultima TV, Rigaku, Japan). Then, the XRD pattern and the reference image of the specimens were analyzed and compared to determine the level of zirconia phase transition.

### 2.6. Statistical Analysis

SPSS 24.0 software was carried out for statistical analysis, and measurement data were expressed as the mean ± standard deviation (mean ± SD). The roughness of each group of specimens was compared using one-way analysis of variance and LSD method. Besides, comparisons between two groups were analyzed by independent samples *t*-test. Enumeration data were expressed as frequency (*n*), and a chi-square test was used for the comparison of multiple groups. *P* < 0.05 was regarded to be significant difference.

## 3. Results

### 3.1. Effects of Different Polishing Systems and Duration on Surface Roughness of Specimens

Effects of different polishing systems and duration on surface roughness of specimens were compared. According to the comparison results, the GR group had the highest roughness; the roughness of specimens polished for 20 s for different polishing systems was significantly higher than those polished for 40 s and 60s for the same polishing systems. However, there was no significant difference in the roughness of the specimens with the polishing duration of 40 s and 60 s between the two polishing systems (Table 2). Subsequently, the roughness of specimens prepared by different polishing systems with the same polishing duration was further compared. The results indicated that the Y 20 and T20 groups were not significantly different, while the roughness of the specimens in both Y 40 and Y 60 groups was significantly higher than that of the T40 and T60 groups (Table 3). The above results revealed that lengthening polishing duration could reduce the surface roughness of the specimens and the surface roughness of the specimens prepared by TOB system was low.

RETRACTED

### 3.2. Influence of Different Polishing Systems on Specimen Surface Morphology

Specimen surface morphology was further analyzed in detail. The analysis results displayed that, in the GL group, the specimens had smooth surface and regular shape and obvious defects were not observed. However, in the GR group, the specimens, with rough surface and irregular shape, were observed wide and deep scratches and dense pits. After polishing, the scratches on the surface of specimens showed a decreasing trend. Moreover, with the increase of polishing duration, the surface morphology was gradually smooth, the shape was regular, and the defects were reduced for the specimens using different polishing systems. Nevertheless, the surface morphology of the Y group was slightly rougher than that of the T group with the same polishing duration (Figure 2).

### 3.3. Influence of Different Polishing Systems and Duration on Crystal Structure of Specimens

Influence of polishing systems and duration on crystal structure of specimens was further investigated. The results showed that, compared with the specimens without grinding and polishing (control), the specimens after grinding and polishing showed the similar XRD model and peak distribution (Figure 3). The above results revealed that, neither application of the occlusion adjustment with carborundum simulation, nor polishing process caused phase transition of zirconia specimens.

## 4. Discussion

Grinding, which can obviously increase the roughness of the restoration surface, is an unavoidable operation in clinical dentistry. Rough restorative surfaces can lead to attachment plaque, opposing tooth wear, and changes in mechanical properties [16]. Appropriate polishing of restorations can improve surface gloss and reduce attachment plaque. In a study by Bollen et al. [17], it was shown that plaque attachment could be effectively reduced when the surface roughness Ra value of the restorations was less than 0.2 *μ*m. The Ra value of tooth enamel roughness is generally in the range of 0.45 *μ*m-0.65 *μ*m, and the surface roughness of restorations close to or lower than the range can be clinically accepted [18]. Polishing is a process that high-speed rotating tools rub the ceramic surface under a certain pressure. Specifically, the cutting action of sharp abrasive particles on the tool surface is utilized to remove surface bulges and shallow materials, thereby smoothing ceramic surface. Most of polishing experiments have shown that appropriate polishing can achieve clinically acceptable roughness on the surface of restorations and can achieve the surface that is similar to or even smoother than glazing [19, 20]. The surface roughness of the specimens prepared by different polishing systems and different duration in this study was within the acceptable range.

RETRACTED

Time is an important factor affecting the polishing effect. On the one hand, short-time polishing cannot complete the whole polishing process or achieve good polishing effect. On the other hand, through long-time polishing which can exert the effect of polishing tools, some studies pointed out that the polishing effect is not directly proportional to the length of polishing duration. Silva et al. [21] studied the polishing effect of each stage of polishing tools in the range of 10 s–50 s and found that most polishing tools could not further improve the polishing effect after 40 s. Vichi et al. [22] suggested that polishing for 60 s was the most effective method to reduce the roughness of CAD/CAM silica/glass-based all-ceramic crowns. Polishing for 60 s can produce a higher luster for silica/glass-based all-ceramic crowns with cracks on the surface, which have the better effect than revitrification after sandblasting and polishing. Hulterström and Bergman [23] conducted a relevant study on the polishing duration of ceramic materials and compared the polishing effect of 30 s, 60 s, 120 s and 180 s. It was considered that the polishing duration of 60 s per stage was the most reasonable in the multistage polishing system, which can obtain the most satisfactory polishing effect. In this experiment, the specimen roughness with the polishing duration of 60 s was the lowest, but still higher than the glazed surface, which may be related to the polishing systems as well as the procedure of the operation process. Additionally, clinically acceptable roughness was achieved at 20 s of polishing, and there was no significant difference in roughness between 40 s and 60 s. The above results were similar to the findings of Silva et al.

A study by Amaya-Pajares et al. [24] showed that roughness did not decrease and remained at a stable level after the polishing reached the certain duration. And the length of duration to reach the lowest roughness value is mainly associated with the polishing tool abrasive particles, binders, and the properties of the polished materials. Excessive extension of polishing duration does not increase the polishing effect but may accelerate the aging of polishing tools due to excessive heat production [25],and cause the transformation of the crystalline phase structure of the surface of zirconia materials [12]. Zirconia has following three allotropic structures: monoclinic phase (m-ZrO_2_), tetragonal phase (t-ZrO_2_), and cubic phase (c-ZrO_2_). The above three crystal phases exist in different temperature ranges and can be interconverted. Specifically, at ambient temperature, zirconia exists mainly as m-ZrO_2_; t-ZrO_2_ can also be present at ambient temperature after binding to an appropriate stabilizer; and t-ZrO_2_ is higher in intensify but smaller in volume than m-ZrO_2_ [2]. When the cracks occurs due to external force, the crystal phase structure of the zirconia material surface will undergo a transition from t phase to m phase. The transition is accompanied by a 3-4% increase in size, favoring resistance to the propagation of deleterious cracks, but may cause unstable residual stresses [26]. During clinical shape adjustment and processing of zirconia, the heat and friction produced locally provide external energy for zirconia crystals, which may cause *m* phase transition [12]. However, no changes in the surface crystal structure were observed in most polishing experiments [5, 27–29], including the researches of Caglar et al. [5]. In the study of Al-Haj Husain et al. [27], it is found that XRD results of samples after polishing showed changes in peak values. However, the authors thought that the changes were caused by stress changes rather than structural changes in the crystalline phase. In the study of Park et al. [29], two zirconia polishing tools were applied, and the polishing process was 8 minutes. It is observed that the maximum proportion of monoclinic phase was increased by 0.03% and 0.09%, and no significant changes occurred in the crystalline phase structure of monolithic zirconia before and after polishing. However, in the study of Mai et al. [26], it was suggested that the crystalline phase structure of zirconia surfaces after polishing using different polishing procedures was different. In this experiment, XRD detection of specimens prepared with different polishing duration revealed that the polishing duration had no effect on the surface crystalline structure of the zirconia.

RETRACTED

However, this study also had some limitations. This study was conducted in vitro, and the specimens used were planar and the polishing was performed on the plane, which could not truly simulate the polishing effect of the tip fossa morphology of intraoral restorations. Moreover, dental ceramic polishing pressure is mostly around 2 N [21], while a strict test was not performed in this study. Besides, Goo et al. [30] suggested that zirconia should be polished using a special zirconia polishing tool and thought that diamond polishing systems was more effective than silicon carbide polishing systems. Mai et al. [26] believed that the application of coarse-grained polishing and medium-grained polishing brushes was the key to achieve smooth surfaces, and commercial polishing systems were needed to be particularly considered in the polishing process. However, polishing results between polishing systems were not compared in this study. Additionally, polishing efficiency of grinding heads was also not conducted comparative analysis. The above limitations are the directions that need to be further explored in future studies.

In future implementation, zirconia materials with larger grain size may cause more roughness due to possible grain pull out during finishing and polishing protocols. Nevertheless, the findings of this study denoted that polishing causes stress on zirconia rather than a phase change in the material itself. Future studies should also focus on mechanical properties of monolithic zirconia after polishing regimens.

## 5. Conclusion

The surface roughness of the specimens can be significantly reduced by glazing, and the polishing effect of TOB zirconia polishing system on domestic zirconia (UPzir Solid Zirconia) is better than that of YOU system. In the three-step polishing process, when polishing duration reaches 60 s at each step, the best polishing effect can be achieved without affecting the crystal phase structure of the specimen surface.

## Figures and Tables

**Figure 1:** Preparation of specimens and X-ray diffractometer (XRD) detection. (a) CAD/CAM software was utilized for the typesetting and design of ST zirconium oxide flap disc. (b) The diffraction pattern of X-ray diffractometer (XRD) detection.

**Figure 2:** SEM observation for surface morphology of specimens prepared with different duration and different polishing systems.

**Figure 3:** The detection of X-ray diffractometer (XRD) for crystal structure of specimens prepared with different polishing systems and different durations.

**Table 1:** Grinding head models and rotational speed parameters of polishing systems.

Manufacturer	Grinding head models (function)	Rotational speed recommendation
Youdent, Wuhan (YOU)	SD021HD (adjacent adjustment of occlusal plane)	7000-15000/min
	RDH056 (flat pre-polishing)	7000-15000/min
	RDH058 (high brightness polishing)	7000-15000/min
Toboom, Shanghai (TOB)	CD2124 (adjacent adjustment of occlusal plane)	15000-20000/min
	RD2124 (flat prepolishing)	10000-15000/min
	RD2125 (high brightness polishing)	8000-12000/min

**Table 2:** Roughness comparison between groups.

Group	*N*	Surface roughness (nm)	*F* value/*P* value
GL	6	38.26 ± 19.17	*F* = 40.944/*P* < 0.001
GR	6	975.97 ± 121.93	
T20	6	544.66 ± 131.46	
T40	6	337.30 ± 23.55	
T60	6	266.94 ± 28.71	
Y20	6	619.27 ± 193.11	
Y40	6	436.54 ± 33.84	
Y60	6	407.97 ± 117.61	

RETRACTED

**Table 3:** Comparison between the same subgroups in Y group and T group.

Group	Surface roughness (nm)	Group	Surface roughness (nm)	Group	Surface roughness (nm)
Y20	619.26 ± 193.11	Y40	436.53 ± 33.84	Y60	407.96 ± 117.61
T20	544.65 ± 131.46	T40	337.30 ± 23.55	T60	266.94 ± 28.71
*T* value	0.782	*T* value	5.896	*T* value	2.853
*P* value	0.455	*P* value	<0.001	*P* value	0.031

## Data Availability

The data used to support the findings of this study are available from the corresponding author upon request.
